# Deep Learning-Based CT Imaging in the Diagnosis of Treatment Effect of Pulmonary Nodules and Radiofrequency Ablation

**DOI:** 10.1155/2022/7326537

**Published:** 2022-08-13

**Authors:** Chengwei Zhou, Xiaodong Zhao, Lili Zhao, Jiayuan Liu, Zixuan Chen, Shuai Fang

**Affiliations:** ^1^Department of Thoracic Surgery, The Affiliated Hospital of Medical School of Ningbo University, Ningbo 315020, China; ^2^Prevention and Health Section, The Affiliated Hospital of Medical School of Ningbo University, Ningbo 315020, China

## Abstract

To study the effect of computerized tomography (CT) images based on deep learning algorithms on the diagnosis of pulmonary nodules and the effect of radiofrequency ablation (RFA), the *U*-shaped fully convolutional neural network (FCNN) (*U*-Net) was enhanced. The convolutional neural network (CNN) algorithm was compared with the *U*-Net algorithm, and segmentation performances were analyzed. Then, it was applied to the CT image diagnosis of 110 lung cancer patients admitted to hospital. The patients in the observation group (55 cases) were diagnosed based on the improved *U*-Net algorithm, while those in the control group (55 cases) were diagnosed by traditional methods and then treated with RFA. The Dice coefficient (0.8753) and intersection over union (IOU) (0.8788) obtained by the proposed algorithm were remarkably higher than the Dice coefficient (0.7212) and IOU (0.7231) obtained by the CNN algorithm, and the differences were considerable (*P* < 0.05). The boundary of the pulmonary nodule can be segmented more accurately by the proposed algorithm, which had the segmentation result closest to the gold standard among the three algorithms. The diagnostic accuracy of the pulmonary nodule in the observation group (95.3%) was superior to that of the control group (90.7%). The long diameter, volume, and maximum area of the pulmonary nodule of the observation group were significantly higher than those of the control group, with substantial differences (*P* < 0.05). Patients were reexamined after one, three, and six months of treatment, and 71 patients (64.55%) had complete remission, 32 patients (29.10%) had partial remission, 6 patients (5.45%) had stable disease, and 1 patient (0.90%) had disease progression. The remission rate (complete remission + partial remission) was 93.65%. The improved *U*-NET algorithm had good image segmentation performance and ideal segmentation effect. It can clearly display the shape of pulmonary nodules, locate the lesions, and accurately evaluate the therapeutic effect of RFA, which had clinical application value.

## 1. Introduction

Today, lung cancer has attracted people's attention with its extremely high incidence. Research data showed that the mortality rate of lung cancer was the first among all cancer deaths, and the incidence and mortality of men were significantly higher than those of women [1]. Most patients with lung cancer have already missed the best treatment time when they are diagnosed. Studies revealed that if it can be diagnosed in advance, the survival rate of early-stage lung cancer patients can reach about 70–80% [2, 3]. Therefore, early diagnosis of lung cancer has become a key issue in improving the cure rate of it. However, the symptoms of the pulmonary nodule in patients with early lung cancer are abnormally subtle, and the manifestation is not obvious, so it is easy to be misdiagnosed and missed by doctors. CT scan diagnosis has become a common and important method of medical diagnosis. Pulmonary nodule is the main feature for judging early lung cancer. It is particularly important to segment the pulmonary nodule completely and finely from the lung image [4]. Traditional medical image segmentation extracts the pulmonary nodule based on the shallow features of the image, which relies on the judgment of the doctor. The addition of subjective factors will lead to inaccurate segmentation. Sivaraj et al. [5] proposed a method of using fuzzy logic technology to determine the threshold to achieve accurate segmentation of melanin, but the segmentation effect was extremely poor, and the efficiency was low.

With the development of artificial intelligence and information, convolutional neural network (CNN) is used in the segmentation of medical images. Cruz et al. [6] proposed and used it in the semantic segmentation of natural images, which made great progress at that time. It surpassed the traditional segmentation method in the past segmentation experience, but its shortcomings are hard to be ignored. The multiplier used in the upsampling operation is too large, resulting in insufficient segmentation accuracy and insufficient fusion of context information, thereby resulting in low accuracy and precision. They have a great impact on the follow-up diagnosis and survival rate post-treatment [7, 8]. However, the birth of the fully convolutional neural network (FCNN) has made a huge contribution to this problem. The *U*-Net network, as a representative of FCNN, can make good use of lower-level information during sampling operations and can merge information at high level [9]. More and more follow-up research combined some good performance network structures with *U*-Net networks. Guo et al. [10] rectified *U*-Net to strengthen the position of the feature map, thereby improving the accuracy of extracting segmentation contours. The 3DU-Net model [11] improved the segmentation performance by learning the spatial information of the image.

Therefore, an algorithm based on the *U*-NET network was proposed in this work, which added residual learning and initial structure and avoided the degradation of network performance while increasing network width and depth. The segmentation performance of the proposed algorithm was compared with the CNN algorithm and the *U*-NET algorithm by applying it to CT images of 110 lung cancer patients. This work aimed at exploring its application value in the evaluation of pulmonary nodules and summarizing the morphological characteristics of pulmonary nodules. This work aimed at improving the effectiveness of radiofrequency ablation (RFA) for patients and laying the foundation for its future clinical application.

## 2. Materials and Methods

### 2.1. Research Objects

In this study, 110 patients with lung cancer admitted to hospital from August 4, 2018 to June 5, 2020 were selected as the research subjects, including 69 males and 41 females, aged between 20 and 80 years. The patients in the observation group (55 cases) were diagnosed based on the improved U-NET algorithm, while patients in the control group (55 cases) were diagnosed using the traditional U-NET algorithm. This study had been approved by the ethics committee of hospital. The patients and their family members knew about this study and signed the informed consent.

#### 2.1.1. Inclusion Criteria

The inclusion criteria are as follows: (i) patients pathologically confirmed as primary lung cancer; (ii) patients with complete clinical data; (iii) patients who had signed the informed consent; and (iv) patients who had not received preoperative radiotherapy or chemotherapy.

#### 2.1.2. Exclusion Criteria

The exclusion criteria are as follows: (i) patients with other malignant tumors; (ii) patients with secondary lung cancer; (iii) patients with complicated mental diseases; (iv) patients who quitted the experiment due to personal reasons; (v) patients with severe cardiovascular and cerebrovascular diseases; and (vi) patients with severe endocrine and metabolic diseases.

### 2.2. Pulmonary Nodule Segmentation Algorithm Based on Improved *U*-Net

The ability of deep learning to extract features is beyond the reach of previous machine learning. Since the *U*-Net network is more capable of processing and fusing high-level and low-level information than CNN, it is widely used in medical image segmentation. To improve the segmentation accuracy of pulmonary nodule images, improvements were made based on the *U*-Net network, and a new pulmonary nodule image segmentation algorithm was constructed.

The *U*-Net network architecture consists of an encoding path and a decoding path. The encoding path can obtain spatial information, which is composed of multiple convolutional layers and downsampling layers. The decoding path can restore the input resolution, performs subconvolution and upsampling of these features, and connects the decoding path and the encoding path through a layer jump connection. The feature information of the high level and the bottom level is combined, and the same weight is given to make it more emphasis on the features of the bottom level. However, due to the small area of the pulmonary nodule image and the varying shape, the accuracy of image segmentation is not high. The batch normalization process is added to the *U*-Net network as follows. The input sample is *a* : *β*={*a*_1_, *a*_2_,…, *a*_*n*_}, and the average of the input sample is as follows:

(1) $$\begin{array}{c} \upsilon_{\beta }=\frac{1}{n}\sum_{i=1}^{n}a_{i}. \end{array}$$

The input sample variance is as follows:

(2) $$\begin{array}{c} \sigma_{\beta }^{2}=\frac{1}{n}\sum_{i=1}^{n}{\left(a_{i}-\upsilon_{\beta }\right)}^{2}. \end{array}$$

According to equations (1) and (2), the input samples are normalized to obtain the distribution data from 0 to 1:

(3) $$\begin{array}{c} a_{i}^{\prime }=\frac{a_{i}-\upsilon_{\beta }}{\sqrt{\sigma_{\beta }^{2}+\gamma }}, \end{array}$$

where *γ* is a very small positive number, and when the divisor is 0, it is calculated by equation (3). The offset is given as

(4) $$\begin{array}{c} b_{i}=\lambda a_{i}^{\prime }+\varepsilon , \end{array}$$

where *b*_*i*_ is the offset, *λ* is the scale factor, and *ε* is the translation factor. After they are added, the problem of low network expression ability can be solved. Due to the increase of neural network levels, there will be performance degradation in the deep network during training. The deeper the network, the more serious the situation. The gradient of the weight *s*_*i*_^1^ of the first layer of the loss function is as follows:

(5) $$\begin{array}{c} \frac{\partial d}{\partial s_{i}^{1}}=\frac{\partial d}{\partial y^{m}}\frac{\partial y^{m}}{\partial y^{m-1}}\frac{\partial y^{m-1}}{\partial y^{m-2}}...\frac{\partial y^{2}}{\partial y^{1}}\frac{\partial y^{1}}{\partial s_{i}^{1}}, \end{array}$$

where *d* is the loss function and *y*^*m*^ is the output of the *m*-th layer. When the range of the first layer is greater than 1 and less than or equal to *m*, the partial conductance of the *m* − 1th layer will be less than 1, which causes the gradient in equation (5) to become exponentially weak. In response to this problem, residual learning is added.

It is supposed that the input is *c*, the output is *h*(*c*), and the residual mapping is *f*(*c*)=*h*(*c*) − *c*. *c* is directly passed to *h*(*c*) by a shortcut, so that it can learn *f*(*c*) directly. The partial derivative of *c* is *y*=*f*(*c*)+*c*:

(6) $$\begin{array}{c} \frac{\partial y}{\partial c}=1+\frac{\partial f\left(c\right)}{\partial c}. \end{array}$$

From the above equation, the partial derivative in the above equation must be greater than 1, so performance degradation will not occur as the network level increases. The residual learning unit is shown in Figure 1.

To increase the width and depth of the network, the Inception [12] network added in this research can keep the computational cost basically unchanged. There are many more convolution kernels and convolution pools of different sizes between input and output, and multiple Inceptions can be merged together, which greatly increases the depth and width. The Inception structure is shown in Figure 2.

The improved *U*-Net network structure is shown in Figure 3.

### 2.3. Extraction of Regions of Interest in Lung CT Images

The purpose of segmenting lung images is classifying pulmonary nodule, but usually, there is a lot of material information in the obtained CT images. Some irrelevant signals will cause a great interference to the segmentation of the pulmonary nodule, so the image needs to be preprocessed. The following method was adopted to extract lung parenchyma. First, the histogram was equalized, and the pixels in the image were redistributed to enhance the contrast of light and dark in each part of the image. Then, the binarization process was performed to calculate the average of the pixels in the image, and the value smaller than the average value was regarded as 0; otherwise, it was regarded as 1. After which, the method of corrosion expansion was used to process the morphology of the image, and pixels were deleted or added at the segmentation boundary to eliminate a certain degree of noise. Finally, the ROI was extracted, and the pulmonary nodule mask was extracted. The pixel of the pulmonary nodule segmentation was 1, and the bright spot was obtained. The remaining part was displayed in black to obtain the result.  Figure 4 shows the specific extraction process.

### 2.4. Simulation

Network parameters: the input image resolution was 256 × 256, the convolution kernel size was 64 × 64 × 64, the learning rate was 0.001, the optimization algorithm was Adam, the number of iterations was 200 epochs, and the loss function was Dice loss.

In this research, the lung CT image data were used as the simulation object, and the CNN algorithm and *U*-Net algorithm were introduced to be compared with the proposed algorithm. The metric index was Dice coefficient [13]:

(7) $$\begin{array}{c} \text{Dice}=\frac{2\left|E\cap F\right|}{\left|E\right|+\left|F\right|}. \end{array}$$

The above equation is the gold standard for pulmonary nodule segmentation, *F* is the segmentation result, and the Dice coefficient has a value range of [0, 1]. The larger the value, the better the algorithm performance. The intersection over union (IOU) in the following equation evaluates the segmentation effect:

(8) $$\begin{array}{c} IOU=\frac{E\cap F}{E\cup F}. \end{array}$$

The larger the value, the more accurate the segmentation. The accuracy and recall rate are calculated as follows:

(9) $$\begin{array}{c} \text{Precision}=\frac{\text{TP}}{\text{TP}+\text{FP}}. \end{array}$$

(10) $$\begin{array}{c} \text{Recall}=\frac{\text{TP}}{\text{TP}+\text{FN}}. \end{array}$$

In equations (9) and (10), TP indicates that the detected pulmonary nodule is true positive, FP indicates that the detected pulmonary nodule is false positive, and FN indicates that the detected pulmonary nodule is false negative.

### 2.5. CT Examination and RFA

128-slice spiral CT machine was employed for diagnosis. Routine bowel preparations were performed before the examination, and scanning was performed after the bladder was properly filled. The patient held the head with both hands, the lower limbs were in the abduction position, and the supine position was in the center of the examination table. The mid-sagittal position of the body was vertical to the plane of the bed, and the head entered advanced. During the examination, the patient should maintain a calm mind, not move his body, and hold his breath as required. The scanning parameters were as follows. The tube voltage was 110 kV, the tube current was 100 mAs, CarekVsemi. United Imaging uCT760: tube voltage was 100 kV, tube current was 80 mAs, with automatic tube current modulation, pitch of 0.938, and lung window filter function B-SHARP-C. The reconstruction layer thickness was 1.5 mm, and the layer spacing was 2.5 mm. The scan range was from the tip of the lung to the bottom of the lung, with both sides including the chest wall and axilla. Lung window was taken for image analysis. Two experienced doctors reviewed the CT images separately, and they reached a conclusion after discussion when their opinions were inconsistent.

The specific procedures of RFA were as follows: (i) the general information of the patients was mastered preoperatively, and fasting and injection of 50 mg pethidine were made. (ii) The basic condition of the tumor was judged according to imaging examination, and the patient's proper lying position was set, so that the focus was closest to the point of entry; it was important to not to pass through the air tube, blood vessel, and other human structures. (iii) With both arms upward, markers were used to locate the puncture area, and a uniform rate of breathing was maintained. Then, it rotated 200° at a speed of 20°/s for scanning. The puncture point was selected according to the mass condition, the surgical area was disinfected, local anesthesia (2% lidocaine) was performed on the skin and chest parietal layer, and the needle was left. (iv) When the needle entered the muscle layer through the anchor point, patients were kept in the state of holding breath. The ablation needle was quickly put down to a certain depth and fixed, and then, the scanning was performed again. It was determined whether the ablation needle was properly located. (v) After it was confirmed that the tip of the ablation needle was in the center of the lesion, the electrode needle was opened and the scanning was performed again to confirm that the electrode needle reached the appropriate position, and then, RFA was performed. (vi) During ablation, the power was 150 W, the temperature slowly rose from 90°C to 103°C, and the time was controlled within 12–23 min. If the tumor was too large, multipoint, multiplanar, and fractional ablations were needed. If the patient felt significant pain during this period, 50 mg pethidine was given. (vi) Scanning was performed again to observe the ablation.

Evaluation of the effect of RFA: (i) complete remission—the tumor disappeared or was smaller than the original 1/4, or there was a cavity in the tumor; (ii) partial remission—the reduction of the tumor's largest diameter was greater than 1/3 of the original size, or the tumor density had changed, showing a tendency of liquidity; (iii) the disease was stable, the largest diameter of the tumor was reduced by less than 1/3 of the original size, or the tumor appeared as a solid; and (iv) the disease progressed. The maximum diameter of the tumor increased by more than 1/5, or the tumor density increased or it invaded adjacent tissues.

### 2.6. Observation Indexes

The number of nodules detected in the two groups of patients was recorded. The accuracy, misdiagnosis rate, and missed diagnosis rate were calculated. The long diameter, short diameter, maximum area, and volume of the pulmonary nodule detected in the two groups of patients were recorded, analyzed, and compared. DAP (cGy·cm^2^) of each RFA of the patient was recorded, and the effective dose was calculated, *ED*=*K* × *DPA*, where *K*=0.14*mSv*/Gycm^2^ was the conversion coefficient.

Follow-up was implemented for RFA. The diagnostic criteria for the efficacy of solid tumors were adopted, and the diagnostic efficacy was classified into four types, including complete remission, partial remission, stable disease, and disease progression, as shown in Table 1. CT review time was set at one month, three months, and six months after ablation.

### 2.7. Statistical Methods

SPSS 22.0 was employed for data statistics and analysis. Mean ± standard deviation ($\bar{x}\pm s$) was how measurement data were expressed, and percentage (%) was how count data were expressed. The difference was statistically considerable with *P* < 0.05.

## 3. Results

### 3.1. Simulation Effects of Three Algorithms

Figure 5 shows the loss curves of the three algorithms. The CNN algorithm started to converge at around 34 iterations, and finally, the loss value was 0.1. The *U*-Net algorithm started to converge at about 20 iterations, and finally, the loss value was 0.7. The convergence speed of the proposed algorithm was obviously much faster than the other two algorithms in the training process, and the final loss value was 0.35.

Figure 6 shows the comparison of the segmentation indexes of the three algorithms. The Dice coefficient (0.8753) obtained by the proposed algorithm was significantly higher than the Dice coefficient (0.7212) obtained by the CNN algorithm, and the IOU (0.8788) was significantly higher than the IOU (0.7231) obtained by the CNN algorithm, with statistically remarkable differences (*P* < 0.05). The precision and recall rate were also higher than the other two algorithms, but there was no significant difference. Referring to the gold standard, each segmentation index of the proposed algorithm was improved, and the segmentation effect of the proposed algorithm was better than the CNN algorithm and the *U*-Net algorithm.

### 3.2. Comparison of CT Image Segmentation Effects of Three Algorithms

Figure 7 shows the comparison of CT image segmentation effects of the three algorithms. Taking the gold standard as a reference, when the CNN algorithm was employed for segmentation, the segmentation effect was very unsatisfactory. It recognized the blood vessels in tissues other than the pulmonary nodule as pulmonary nodule and separated them. When the *U*-Net algorithm was used for segmentation, the segmentation results were obviously much better, but there was a bit of suspicion of excessive segmentation. When the proposed algorithm was used for segmentation, the boundary of the pulmonary nodule was segmented more accurately, and the segmentation result was the closest to the gold standard among the three algorithms.

### 3.3. Comparison of the Detection of Pulmonary Nodule between the Two Groups

Figure 8 shows the comparison of the accuracy and misdiagnosis rate of the pulmonary nodule in the two groups. A total of 1,120 lesions were distributed among 110 patients. There were lesions in upper lung (511 cases), accounting for 45.6%, followed by the lower lung (372 cases), accounting for 33.2%, and the middle lung (237 cases), accounting for the least, which was 21.2%; 753 nodules were detected in the control group, 70 were misdiagnosed, the accuracy was 90.7%, and the misdiagnosis rate was 9.3%. In the observation group, 1,126 nodules were detected and 53 were misdiagnosed. The accuracy was 95.3%, and the misdiagnosis rate was 4.7%.

### 3.4. Comparison of Pulmonary Nodule Long Diameter and Short Diameter between Two Groups of Patients

Figure 9 shows the comparison of the pulmonary nodule long diameter between the two groups. The long diameter of the pulmonary nodule (21.6 ± 1.5 mm) of the observation group was significantly higher than that of the control group (13.1 ± 0.67 mm), with substantial differences (*P* < 0.05).

Figure 10 shows the comparison of the pulmonary nodule short diameter between the two groups. The difference between the short diameter of the pulmonary nodule (2.4 ± 1.07 mm) of the observation group and that of control group (2.6 ± 1.2 mm) was not remarkable (*P* > 0.05).

### 3.5. Comparison of the Maximum Area and Volume of Pulmonary Nodule between Two Groups of Patients

Figure 11 shows the comparisons of the pulmonary nodule volume and maximum area of the two groups of patients. The maximum area of the pulmonary nodule in the observation group (261.3 ± 50.4 mm^2^) was significantly higher than that of the control group (107.5 ± 50 mm^2^). The volume of pulmonary nodule (2257.6 ± 400 mm^3^) was also significantly higher than that of the control group (654.7 ± 201 mm^3^), and the difference was statistically significant (*P* < 0.05).

### 3.6. RFA Effect

Figure 12 shows the comparison of the cumulative and effective doses of RFA between the two groups. The cumulative dose of RFA in the observation group (172.3 ± 45.3 mGy) was significantly higher than that in the control group (83.4 ± 30.2 mGy). The effective dose of RFA (5.34 ± 1.21 mSv) was significantly higher than that of the control group (2.53 ± 0.94 mSv), with significant differences (*P* < 0.05).  Figure 13 shows the efficacy evaluation of 110 patients after RFA. After 1, 3, and 6 months of treatment, 71 cases (64.55%) had complete remission, 32 cases (29.10%) had partial remission, 6 cases (5.45%) were stable, and 1 case (0.90%) had disease progression. The remission rate (complete remission + partial remission) was 93.65%. The area of the lesion area oozed out from the blur, the surrounding fiber strands were formed, and the nodules at the lesion area disappeared.

## 4. Discussion

Lung cancer affects people's quality of life and physical health and has an extremely high incidence, and it ranks first among many cancer deaths, accounting for 17.5% of cancer deaths [14]. In recent years, people have paid more and more attention to health, and CT imaging plays a very important role in detecting cancer. The accuracy and resolution requirements of the image are extremely high. With the rapid development of artificial intelligence and informatization, the application of deep learning in medical imaging has made great contributions to the segmentation and diagnosis of medical images [15]. In this research, the *U*-Net algorithm was improved and compared with the CNN algorithm and the *U*-Net algorithm. The results showed that the CNN algorithm started to converge at about 34 iterations, and the final loss was about 0.1. The *U*-Net algorithm started to converge at about 20 iterations, and the final loss was about 0.7. The convergence speed was obviously much faster than the other two algorithms in the training process of the proposed algorithm, and the final loss was about 0.35. The Dice coefficient (0.8753) and IOU (0.8788) obtained by the proposed algorithm were significantly higher than the Dice coefficient (0.7212) and IOU (0.7231) obtained by the CNN algorithm, and the differences were statistically substantial (*P* < 0.05). In addition, the precision and recall rate were also higher than the other two algorithms, and there was no significant difference. It showed that referring to the gold standard, the proposed algorithm had better image segmentation performance while retaining edge and detail information [16].

After that, the improved *U*-Net algorithm was applied to the CT image diagnosis of 110 lung cancer patients admitted to hospital. The results showed that there were 1,120 lesions in 110 patients, 511 cases in the upper lung, accounting for 45.6%, 372 cases in the lower lung, accounting for 33.2%, and 237 cases in the middle lung, accounting for 21.2%. The control group had 753 nodules detected and 70 nodules misdiagnosed, the accuracy rate was 90.7%, and the misdiagnosis rate was 9.3%. The observation group had 1,126 nodules detected and 53 nodules misdiagnosed, the accuracy was 95.3%, and the misdiagnosis rate was 4.7%. It showed that visual fatigue may occur during manual reading, and the blood vessels next to the pulmonary nodule were misdiagnosed as pulmonary nodule. The addition of the proposed algorithm greatly improved the accuracy of medical image diagnosis of patients with pulmonary nodule and reduced the risk of missed diagnosis. It was consistent with the results of Schwyzer et al. (2020) [17]. The long diameter (21.6 ± 1.5 mm), volume (2257.6 ± 400 mm^3^), and maximum area (261.3 ± 50.4 mm^2^) of the pulmonary nodule of the observation group were significantly higher than the long diameter (13.1 ± 0.67 mm), volume (654.7 ± 201 mm^3^), and maximum area (107.5 ± 50 mm^2^) of the control group. The differences were statistically significant (*P* < 0.05). However, the short diameter of the pulmonary nodule (2.4 ± 1.07 mm) was not statistically significant (*P* > 0.05) compared with the control group (2.6 ± 1.2 mm). This may be closely related to the characteristics of the tumor. It not only invaded the surrounding tissues of the tumor, but also increased rapidly, which was similar to the results of Mulshine et al. [18]. Studies showed that the addition of the proposed algorithm had many advantages in detecting the volume, area, and length of the pulmonary nodule and was suitable for the detection of early lung cancer. In addition, the prediction of malignant nodules was accurate. Finally, RFA was performed on the two groups of patients to compare the cumulative dose and effective dose of radiation between the two groups. The results showed that the cumulative dose and effective dose of RFA in the observation group ((172.3 ± 45.3 mGy) and (5.34 ± 1.21 MSV)) were significantly higher than those in the control group ((83.4 ± 30.2 mGy) and (2.53 ± 0.94 MSV), and the differences were statistically significant (*P* < 0.05). Patients were reexamined after one, three, and six months of treatment, and 71 patients (64.55%) had complete remission, 32 patients (29.10%) had partial remission, 6 patients (5.45%) had stable disease, and 1 patient (0.90%) had disease progression. The remission rate (complete remission + partial remission) was 93.65%. This was consistent with the research results of Dornbusch et al. [19]. The addition of deep learning algorithms made the diagnosis and segmentation of patient pulmonary nodule more accurate, which effectively helped medical staff identify the lesion and then accurately ablated it to achieve ideal treatment results.

## 5. Conclusion

The *U*-Net algorithm was improved and compared with the CNN algorithm and *U*-Net algorithm, and then was applied to the CT image diagnosis of 110 lung cancer patients. The results showed that the network of the proposed algorithm had better image segmentation performance among all algorithm, and the segmentation effect was good. The addition of the proposed algorithm made the diagnosis operation of CT images simple and accurate in medical diagnosis. The shape of the pulmonary nodule was clearly displayed to the medical staff. In addition, it also had a precise positioning effect for the follow-up RFA, which realized an ideal treatment effect. However, due to limited conditions, the sample size included in this work was small and the study duration was short, so it was necessary to continue to expand the sample size and increase the study duration to explore the long-term therapeutic effect. In conclusion, CT images based on the deep learning algorithm could provide a reference for the diagnosis of pulmonary nodules and the subsequent research on the therapeutic effect of RFA, which showed high clinical application value.

## Figures and Tables

**Figure 1:** Residual learning unit.

**Figure 2:** Inception structure.

**Figure 3:** Improved *U*-Net network model.

**Figure 4:** Extraction process.

**Figure 5:** Loss curves of the three algorithms.

**Figure 6:** Comparison of the segmentation indicators of the three algorithms. ^*∗*^Compared with the CNN algorithm, *P* < 0.05.

**Figure 7:** Comparison of CT image segmentation effects of three algorithms. (a) The original image; (b) the pulmonary nodule; (c) the gold standard; (d) the CNN's segmentation result; (e) *U*-Net's segmentation result; (f) the proposed algorithm's segmentation result.

**Figure 8:** Comparison of the accuracy and misdiagnosis rate of the pulmonary nodule in the two groups of patients. (a) Control group and (b) observation group.

**Figure 9:** Comparison of the pulmonary nodule long diameter between two groups of patients. ^*∗*^Compared with the control group, *P* < 0.05.

**Figure 10:** Comparison of the pulmonary nodule short diameter between two groups of patients.

**Figure 11:** Comparison of the maximum area and volume of the pulmonary nodule between the two groups. ^*∗*^Compared with the control group, *P* < 0.05.

**Figure 12:** Comparison of cumulative dose and effective dose of RFA between the two groups. ^*∗*^Compared with the control group, *P* < 0.05.

**Figure 13:** Evaluation of the curative effect of patients after RFA.

**Table 1:** Diagnostic criteria for the efficacy of solid tumors.

Clinical efficacy	Nodule size	Nodule density	PET
Complete remission (two)	Lesions disappeared <25% before treatment	Small vacuole formation	Standard uptake value (SUV) <2.5
Partial remission (one)	Maximum diameter reduction ≥30% before treatment	Low-density changes of the lesion, necrosis of the central part	Decreased SUV
Stable disease (one)	Maximum diameter reduction <30% before treatment	Characteristic manifestations of solid tumors, without central necrosis	Unchanged SUV
Disease progression (two)	Maximum diameter increase ≥20% before treatment	Features of solid tumors, invasion of adjacent tissues	Increased SUV

## Data Availability

The data used to support the findings of this study are available can be obtained from the corresponding author upon request.
